This article has been retracted.

# Suitable nitrogen application mode and lateral spacing for drip-irrigated winter wheat in North China Plain

**DOI:** 10.1371/journal.pone.0260008

**Published:** 2021-11-12

**Authors:** Muhammad Zain, Zhuanyun Si, Jinsai Chen, Faisal Mehmood, Shafeeq Ur Rahman, Adnan Noor Shah, Sen Li, Yang Gao, Aiwang Duan

**Affiliations:** 1 Key Laboratory of Crop Water Use and Regulation, Ministry of Agriculture and Rural Affairs /Institute of Farmland Irrigation, Chinese Academy of Agricultural Sciences, Xinxiang, Henan, PR China; 2 Graduate School of Chinese Academy of Agricultural Sciences, Beijing, PR China; 3 Faculty of Agricultural Engineering, Sindh Agriculture University, Tandojam, Pakistan; 4 Department of Agricultural Engineering, Khwaja Fareed University of Engineering and Information Technology, Rahim Yar Khan, Punjab, Pakistan; Institute of Genetics and Developmental Biology Chinese Academy of Sciences, CHINA

## Abstract

To propose an appropriate nitrogen application mode and suitable drip irrigation lateral spacing, a field experiment was conducted during 2017–2018 and 2018–2019 growing seasons to quantify the different drip irrigation lateral spacings and nitrogen fertigation strategies effects on winter wheat growth, yield, and water use efficiency (WUE) in the North China Plain (NCP). The experiment consisted of three drip irrigation lateral spacing (LS) (40, 60, and 80 cm, referred to as D_40_, D_60,_ and D_80_ respectively) and three percentage splits of nitrogen application modes (NAM) (basal and top dressing application ratio as 50:50 (N_50:50_), 25:75 (N_25:75_), and 0:100 (N_0-100_) respectively). The experimental findings depicted that yield and its components, and WUE were markedly affected by LS and NAM. Fertigation of winter wheat at N_25:75_ NAM notably (P<0.05) increased the grain yield by 4.88%, 1.83% and 8.03%, 4.61%, and WUE by 3.10%, 3.18% and 5.37%, 7.82%, compared with those at NAM N_50:50_ and N_0:100_ in 2017–2018 and 2018–2019 growing seasons, respectively. LS D_40_ appeared very fruitful in terms of soil moisture and nitrogen distribution, WUE, grain yield, and yield components than that of other LS levels. The maximum grain yield (8.73 and 9.40 t ha^-1^) and WUE (1.70 and 1.95 kg m^-3^) were obtained under D_40_N_25:75_ during both growing seasons, which mainly due to that all main yield components in D_40_N_25:75_ treatment, such as spikes per unit area, 1000-grain weight, and grains per spike were significantly higher as compared to other treatments. The outcomes of this research may provide a scientific basis of lateral spacing and nitrogen fertigation management for the production of drip-irrigated winter wheat in NCP.

## 1. Introduction

Making availability of energy, food resources, and water to the rising world population is a serious challenge. These challenges are chronic in critical regions where food demand is high, and water resources are less. Globally, water scarcity in arid and semi-arid areas is a major concern for agricultural authorities. Sustainable groundwater management in North China is a fundamental challenge, where more than 70% of freshwater is utilized for agricultural purpose [1]. Currel et al. [2] stated that groundwater level in North China Plain (NCP) is decreasing by 0.5–3 m year^-1^ since last three to four decades.

High-performance irrigation systems, like drip irrigation systems, are often encouraged to overtake this problem and to dramatically enhance the irrigation efficiency over traditional irrigation systems. Drip irrigation provides uttermost water productivity by keeping soil moisture at 50–60% field capacity [3]. Tayel and Mansour [4] stated that drip irrigation is among the best water-saving irrigation systems and it has high WUE and fertilizer use efficiency. Nie et al. [5] make a comparison of drip irrigation with surface irrigation and stated that drip irrigation reduced the water consumption of about 57.5–86.4 mm and resulted in an increase in WUE by 6.2–16.0% than that of the surface irrigation method. Wang et al. [3] found that in Daxing, Beijing region, drip irrigation saves about 45.9–114.8 mm water and resulted in 5–13% yield improvement and a significant increase in WUE in winter wheat as compared to level-basin irrigation.

Nitrogen (N) is an essential crop nutrient, that has extreme effects on crop growth and yield [6]. Wei et al. [7] stated that improper management guidance gives rise to the application of N fertilizer by most of the farmers on their own experience the base, without considering the environmental consequences. Globally, we are applying immoderate N and >50% of N is lost to the environment which causes environmental pollution [8]. Liu et al. [9] and Ju et al. [10] reported that ammonia volatilization, denitrification, and nitrate-nitrogen leaching caused 15–45% fertilizer loss in the NCP. It results in dangerous effects on the environment like nitrate-nitrogen leaching and agricultural non-point source pollution in the groundwater. Thus, there is a high need for an efficient fertilization application in this region.

In many cases, soil water and nitrate contents show an interactive effect on the crop yield [11]. Gasser et al. [12] stated that soil nutrient distribution differs in drip irrigation than that of the conventional irrigation method, and it mainly depends on fertilizer application methods, and variations in water movement. Drip fertigation is considered as the advanced technology for saving fertilizer inputs, and has high crop yields by directly delivering the nutrients and water to root zones [13]. Drip fertigation enhanced the tea yield by 1.4% and fertilizer savings of up to 67% as compared to the traditional fertilizer application [14]. Feng et al. [15] demonstrated that 72% of the traditional fertilizer dose by drip fertigation could achieve high water productivity, partial factor productivity, and high potato yield in sandy soils. Zhang et al. [16] and Zhou et al. [17] stated that an adequate amount of water along with a sufficient amount of nutrients can be supplied by drip fertigation throughout the growing season.

In order to properly manage the drip irrigation system, the uniform moisture and fertilizer distribution around the emitters must be apprehended to uniformly wet the crop root zone, which will increase the water/fertilizer use efficiency. In designing drip irrigation systems, the shape of wetted volume and soil moisture distribution within this volume are the two main factors in determining emitter and drip irrigation lateral spacings to obtain uniform water distribution in the root zone. The evenness of soil moisture distribution is based on drip irrigation lateral spacings and on other drip irrigation approaches like irrigation amount and pressure during irrigation, outlet design of drip tubes, and the interval between irrigations [3, 18]. Though, field studies based on drip irrigation needs to be performed to determine the suitable basal: top dressing ratio of nitrogen and drip irrigation lateral spacing which can be helpful for sustainable winter wheat production.

Proper irrigation scheduling is very important for better crop production. Although, an extensive work on irrigation scheduling for winter wheat production has been done in this area [19–21]. But, the information on nitrogen application modes under varying drip irrigation lateral spacings especially in winter wheat is still not documented. Thus, the study was intended to: (i) reveal the movement and distribution of water and nitrogen as affected by different lateral spacings and nitrogen application modes (NAMs); (ii) quantify the growth, yield, and WUE of winter wheat under different drip irrigation lateral spacings; (iii) to investigate the suitable lateral spacings and basal: top dressing ratio of nitrogen for sustainable wheat production in NCP. The outcome of this study will be beneficial for farmers to establish the optimal drip irrigation system for winter wheat in the NCP.

## 2. Material and methods

### 2.1. Site description and climatic condition

The field study was carried out during two consecutive growing seasons (2017–2018 and 2018–2019) of winter wheat at Qiliying Experimental Station (35˚08’N, 113˚45’E; altitude 81 m), Institute of Farmland Irrigation, Chinese Academy of Agricultural Science (CAAS) in Xinxiang, Henan in NCP. The soil characteristics for 0–100 cm of soil layers are described in Table 1. Soil texture was classified as sandy loam, having 1.10% organic matter, 8.5 pH, and electrical conductivity of 257.6 μs cm^-1^. The available (average of 0–100 cm soil layer) soil nitrogen contents were 40.20 mg kg^-1^, phosphorous contents were 11.90 mg kg^-1^, and the potassium contents were 100.51 mg kg^-1^.

**Table 1:** Physical and chemical properties of the experimental field.

Soil layer (cm)	Sand (%)	Silt (%)	Clay (%)	Soil texture	B.D. (g cm^-3^)	Field Capacity (cm^3^ cm^-3^)	Residual water content (cm^3^ cm^-3^)
**0–20**	53.06	43.14	3.80	Sandy Loam	1.56	0.341	0.163
**20–40**	47.96	45.43	6.61	Loam	1.58	0.308	0.157
**40–60**	45.61	48.33	6.06	Sandy Loam	1.54	0.327	0.181
**60–80**	47.96	47.49	4.55	Sandy Loam	1.42	0.283	0.181
**80–100**	81.48	16.95	1.57	Loamy Sand	1.45	0.294	0.173
**Average**	**55.21**	**40.27**	**4.52**	**Sandy Loam**	**1.51**	**0.311**	**0.171**

Note: B.D. is Bulk density.

The meteorological data on daily basis including air temperature (maximum and minimum), relative humidity, solar radiation, wind velocity, precipitation, and air pressure was recorded from the automatic weather station installed at the experimental site. According to meteorological data, the seasonal rainfall (mid-October to early June) ranged between 60 to 200 mm with average air temperature in-between 10 to 12°C during the winter wheat growing season. However, approximate water consumption of winter wheat is ranged from 450 to 500 mm during the whole growing season [22]. During the growing season of 2017–2018 and 2018–2019, the total precipitation was 238 mm and 117 mm correspondingly. Daily based weather data including precipitation, and minimum and maximum air temperature over the two study years is presented in Fig 1.

**Fig 1:** Precipitation and daily maximum, minimum temperature over the winter wheat growing season in 2017–2018 and 2018–2019.

### 2.2. Experimental design, crop management, and irrigation system

The experimental design was split design with drip irrigation lateral spacings in the main plot, and nitrogen application mode treatments as subplot respectively. The experiment had nine treatments with three replications of each treatment, having a sub-plot size of 3 m × 20 m. Three drip irrigation lateral spacings (LS) were set and referenced as D_40_, D_60,_ and D_80_ with lateral drip tube spacings of 40, 60, and 80 cm respectively. There were three nitrogen application mode (NAM) treatments on the base of basal and top dressing ratios; N_50:50_ (50% application at basal and remaining 50% as top dressing), N_25:75_ (25% application at basal, and remaining 75% as top dressing) and N_0:100_ (all of N as top dressing). The basal dose was broadcasted during bed preparation and the top dressing (at returning green, jointing, and grain filling stage) was carried out by fertigation (Table 2). Shen et al. [23] recommended 36 to 45 mm irrigation quota for high production of winter wheat in the experimental area. In this study, irrigation scheduling was done according to local recommendation by Shen et al. [23], on the basis of accumulative soil water consumption (ASWC), and 50 mm irrigation was performed whenever ASWC reaches 50 mm (Table 2). Furthermore, in several cases 10 mm irrigation was carried out during the 2017–2018 growing period for applying nitrogen fertilizer, even no irrigation was required, and this irrigation amount was subtracted from the scheduled amount for next irrigation in the same treatment [24].

**Table 2:** Irrigation scheduling and fertigation for all treatments during the 2017–2018 and 2018–2019 wheat season.

Year	Date (Day of the Year)	Irrigation (mm)	Fertigation (%)		
			N_50:50_	N_25:75_	N_0:100_
**2017–2018**	287 (2017)	-	50	25	0
	71	50	16.67	25	33.33
	98*	10	16.67	25	33.33
	126**	40	-	-	-
	133*	10	16.67	25	33.33
	287 (2018)	-	50	25	0
**2018–2019**	71	50	16.67	25	33.33
	93	50	16.67	25	33.33
	123	50	-	-	-
	136	50	16.67	25	33.33

Note

*During the 2017–2018 growing season, 10 mm water was irrigated for applying fertilizer even if no irrigation required

** indicates that 10 mm irrigation amount was deducted from designed irrigation treatment for next irrigation scheduling.

On 15 October in both 2017 and 2018, winter wheat cultivar “Zhoumai 22” was planted with 180 kg ha^-1^ seed rate at 20 cm of row spacing. Zhoumai 22 is the dominant variety in the southern region of North China Plain. It has good cold resistance and lodging resistance. Under normal growth, the plant height is about 80 cm, the number of grains per panicle are 36.0, and the 1000 grain weight is 45.4 g. The nitrogen as urea, phosphorous as calcium superphosphate, and potassium as potassium sulfate was applied at the rate of 270, 105, and 120 kg ha ^-1^, respectively. The nitrogen fertilizer was applied according to experimental design as basal and as top dressing at returning green, jointing, and grain filling stage, while all of the phosphorous and potassium fertilizer doses were applied as basal. The top dressing was done with fertigation by dissolving the urea in water until complete dissolution and then added to fertilizer tanks. The harvesting of experimental plots was done on May 31, 2018, and on June 3, 2019, respectively.

The underground pipelines for irrigation purposes were installed at the experimental site. These pipelines were interlinked to pumps, having pressure controllers to maintain the groundwater pressure level. Polyethylene (PE) drip irrigation laterals of 16 mm diameter working at 0.1–0.15 MPa operating pressure were installed in the field. The emitter spacing and discharge rates were 20 cm and 2.2 L h^-1^ respectively. The water flow meter to monitor the exact supply of irrigation was installed at the sub-pipeline of each plot.

Generally, farmers in NCP irrigate the winter wheat on the basis of soil moisture status at returning green stage in early spring [25]. Taking into account this schedule, the first irrigation was done on the same date for all treatments. Whereas the next irrigation was scheduled on the base of ASWC according to experimental design as mentioned above. The quantity and timing of irrigation scheduling and nitrogen fertilizer application during both growing seasons is depicted in Table 2.

### 2.3. Measurements

#### 2.3.1. Growth and yield-related parameters

The growth of winter wheat was characterized by leaf area index (LAI) and average plant height. LAI and plant height of winter wheat was recorded at 10 to 15 days interval from 10 randomly collected plant samples for each sub-plot. LAI was determined according to Jha et al. [19]. According to this method, leaf length and leaf width of each leaf from 10 plants were measured with a ruler, and the following equation was used to calculate leaf area per plant (LA) and is presented in m^2^:

$$LA=\frac{\sum_{i=1}^{n}A_{i}}{n}=\frac{\sum_{i=1}^{n}\left[\sum_{j=1}^{m}(L_{j}\times W_{j})\times 0.8\right]}{n}$$ (1)

LAI was set as a ratio of total leaf area to land area over the experimental plot.

$$LAI=\frac{LA\times N}{S}$$ (2)

where, n is a number of plant samples used to determine leaf area, n = 10; A_i_ is leaf area of i^th^ plant; m is a number of leaf in the i^th^ plant, while L_j_ and W_j_ is length and width of the j^th^ leaf in the i^th^ plant (both calculated in cm); N represents the number of plants (including tillers) in 1 m of the row, and S is row spacing (S = 0.2 m).

Plant height was measured with 10 plants and presented as the mean of the heights from the ground surface to the top of the canopy during initial growth phases and from the ground surface to the topmost of the spikelet (without awns) after the earring stage. At harvest, 10 plants were chosen in each sub-plot to assess plant height, yield components like the number of grains per spike and spike length. Finally, a 1 m^2^ area of plants was sampled to quantify a number of spikes per unit area, 1000-grain weight (g), and grain yield (t. ha^-1^) for each experimental sub-plot. Rubbing and sorting of harvested plants were done by hand. The grain yield of each experimental sub-plot was measured by weighting grains after naturally drying to 12% moisture content.

#### 2.3.2. Evapotranspiration, water use efficiency, and grain yield

To assess the soil moisture and nitrogen content, soil samples were excavated after 5 days of an irrigation event at soil layer of 0–10, 10–20, 20–30, 30–40, 40–60, 60–80, and 80–100 cm in each sub-plot by the auger. The soil samples were collected at 0, 10, and 20 cm to drip lateral in D40, at 0, 15, and 30 cm to drip lateral in D60, and at 0, 20, 40 cm to drip lateral in D80 plots. Each sample was equally divided into two sub-samples to measure the soil moisture and soil nitrogen content. Electronic weight balance was used to assess the weight of one sub-samples to an accuracy of 0.01 g and was oven-dried at the temperature of 105°C for 24 h. The remaining sub-samples were used to measure soil nitrogen (NO_3_^-^). The concentration of soil nitrogen was measured by extracting soil samples for one hour with 2 M KCl (1:10) and then passing through the process of filtration with a 0.45 mm membrane. Then, the soil nitrogen concentrations were determined by using an Auto Analyzer (Seal Analytical Inc. AA3-HR USA).

The soil water balance equation (Eq (3)) was used to determine crop evapotranspiration as used by Chen et al. [26]:

ETc=I+P+U−(R+D)±ΔS (3)

where, I and P are applied irrigation amount and precipitation, respectively; ΔS is a change in the stored soil water in 0–100 cm soil profile, U is the upward flow of groundwater into the root zone, while D and R are downward drainages and surface runoff respectively. Here, upward groundwater flow, downward drainage, and surface runoff were ignored because no heavy rainfall occurred to cause runoff. The irrigation amount was small and the water storage capacity of the study site was high that avoid deep drainage and upward flow.

Accumulative Soil water consumption (ASWC) was calculated by the equation as given below:

ASWC=Soilmoistureafternearestirrigation–Currentlymeasuredsoilmoisture (4)

Water use efficiency (kg.m^-3^) gives evidence of efficacious consumption of an irrigation unit for enhancing crop production. WUE of grain yield (Y, kg.m^-2^) was calculated according to El-Rahman [27].


$$WUE=\frac{Y}{ETc}$$ (5)

### 2.4. Statistical analysis

All collected experimental data was statistically analyzed by using Statistics 8.1 software under a split-plot design with three replications. Analysis of variance (ANOVA) was done to evaluate mean and interaction terms of lateral spacings and nitrogen application mode treatments. Furthermore, the means of different treatments were compared by the least significant difference (LSD) at 5%, 1%, and 0.1% probability levels.

## 3. Results

### 3.1 The movement and distribution of water and nitrogen under different LS and NAMs

#### 3.1.1 Effects of LS and NAM on water movement and distribution

The temporal variations in soil moisture content as influenced by different lateral spacings and NAM during the two wheat-growing seasons are given in Figs 2 and 3 respectively. The variation in soil moisture distribution was significantly influenced by different treatments. The relative soil moisture contents were higher in all plots at the winter wheat re-greening stage, while as the water consumption increased with plant growth, soil moisture contents start decreasing gradually especially after the stem-elongation stage. However, soil moisture was more at later growth stages of wheat during the 2018 growing season because of rainfall events. Higher soil moisture contents were observed under D_40_ as compared to D_60_ and D_80_ lateral spacings during the whole growing season. Under all lateral spacings and nitrogen fertigation treatments, variations in soil moisture at shallow and deepest layers was more prominent i.e., soil moisture contents were higher in 0–10 and 80–100 cm layers and lower moisture contents were at 20–80 cm soil depth. Compared to the D_60_ and D_80_ treatment, D_40_ distributed more water in the deeper soil layer. Surprisingly, declined soil moisture was observed at 30–70 cm depth in all treatments during the whole growing season.

**Fig 2:** Soil moisture (m^3^/m^3^) of various LS and NAMs treatments during the 2018 wheat growing season.

**Fig 3:** Soil moisture (m^3^/m^3^) of various LS and NAMs treatments during the 2019 wheat growing season.

#### 3.1.2 Effects of LS and NAM on nitrate-nitrogen movement and distribution

The temporal variations in soil nitrate-nitrogen due to lateral spacings and nitrogen management treatments are presented in Figs 4 and 5. The figures indicated that soil *NO*_*3*_^*—*^*N* contents at different depths was significantly affected due to lateral spacings and nitrogen treatments during both growing seasons. Comparing the different lateral spacings, higher nitrogen contents were noticed in D_40_ plots than that of D_60_ and D_80_ treatments during both growing seasons. The soil *NO*_*3*_^*—*^*N* contents at the wheat re-greening stage in the 60–100 cm soil layer were higher in treatments with more basal nitrogen as compared to the N_25:75_ and N_0:100_ treatment. In addition, soil *NO*_*3*_^*—*^*N* contents during both growing seasons at D_40_N_0:100_ were markedly higher than other treatments. At the jointing stage, *NO*_*3*_^*—*^*N* contents in the 40–60 cm soil layer of all treatments were decreased and the difference among treatments was smaller. Following the nitrogen application as fertigation at the jointing stage and grain filling stage, soil *NO*_*3*_^*—*^*N* contents of N_25:75_ and N_0:100_ were notably higher than that of N_50:50_ treatment at anthesis and maturity stage respectively.

**Fig 4:** Soil NO3—N contents of various LS and NAMs during the 2018 wheat growing season.

**Fig 5:** Soil NO3—N contents of various LS and NAMs during the 2019 wheat growing season.

### 3.2. Effects of different LS and NAM on crop growth

The data presented in Figs 6 and 7 showed the growth characteristics (LAI and plant height) of winter wheat during the 2018 and 2019 growing seasons respectively. Generally, both the growth characteristics showed almost similar trends under different LS and NAMs in both study seasons. Under all NAMs, plants in D_40_ grew better as opposed to D_60_ and D_80_ during both growing seasons. At earlier growth stages (returning green and tillering), the higher LAI and plant height was observed under N_50:50_ followed by N_25:75_, but at lateral stages (jointing, booting, anthesis) wheat plants under N_50:50_ treatment grew poorly and displayed higher growth at N_0:100_ as compared to the N_25:75_. This indicates that applying more nitrogen was beneficial for wheat LAI and plant height irrespective of the growth stage. The highest values of LAI were observed at the booting stage under all LS and NAMs and then LAI starts decreasing till harvesting during both seasons. The highest values of LAI were recorded in D_40_N_0:100_ while the lowest values were observed in D_80_N_50:50_ during both seasons.

**Fig 6:** Leaf area index of winter wheat in (a) D_40_, (b) D_60,_ and (c) D_80_ during the 2017–2018 and 2018–2019 growing season.

**Fig 7:** Plant height of winter wheat in (a) D_40_, (b) D_60,_ and (c) D_80_ during the 2017–2018 and 2018–2019 growing season.

### 3.3. Effects of different LS and NAM on yield and its components

Drip irrigation lateral spacing and nitrogen application modes both executed highly significant effects on the grain yield. Their interaction showed effects at P < 0.05 significance level during both study seasons (Table 3). A consistent declining trend in grain yield was observed with an increase in drip irrigation lateral spacing during both years. Grain yield ranged from 7.29–8.73 and 7.84–9.40 t ha^-1^ during the growing season of 2017–2018 and 2018–2019, respectively. The highest grain yield (8.73 and 9.40 t ha^-1^) was achieved under D_40_N_25:75_ treatment, while the minimum grain yield (7.29 and 7.84 t ha^-1^) was recorded in D_80_N_50:50_ during both seasons, respectively. Among three drip irrigation lateral spacings, grain yield on D_40_ was highest followed by D_60,_ and was lowest D_80_ during both study seasons. Averaged across the drip irrigation lateral spacings, grain yield was significantly enhanced by increasing top-dressed nitrogen percentage from 50 to 75% but decreased by adding all the nitrogen as top dressing in N_0:100_ treatment.

**Table 3:** Statistics analysis results of winter wheat grain yield (t ha^-1^) during 2017–2018 and 2018–2019 growing season.

Season	2017–2018				2018–2019			
Treatment	N_50:50_	N_25:75_	N_0:100_	Average	N_50:50_	N_25:75_	N_0:100_	Average
**D**_**40**_	8.51	8.73	8.60	**8.61a**	8.87	9.40	9.04	**9.10a**
**D**_**60**_	7.96	8.30	8.14	**8.14b**	8.36	8.99	8.64	**8.66b**
**D**_**80**_	7.29	7.89	7.73	**7.64c**	7.84	8.69	8.21	**8.25c**
**Average**	**7.92c**	**8.31a**	**8.16b**	**8.13**	**8.36c**	**9.03a**	**8.63b**	**8.67**
**Statistics Analysis Results**	**D**	***			**D**	**		
	**N**	***			**N**	***		
	**D × N**	*			**D × N**	*		

D = Drip irrigation lateral spacing, N = Nitrogen basal top dressing ratios. Average values indicating different letters are significantly different at P<0.05. Significance level

*(P < 0.05)

**(P < 0.01)

***(P < 0.001).

Across the two years study data, drip irrigation lateral spacing and nitrogen application modes affected the grain yield components (spike length, number of grains per spike, number of spikes per unit area, and thousand-grain weight) but their interaction was non-significant except for the number of grains per spike during both growing seasons (Table 4). Generally, increasing the drip irrigation lateral spacing resulted in a consistent decrease in yield components. Average across the NAM, D_80_ reduced the spike length, number of grains per spike, number of spikes per unit area, and thousand-grain weight by 5.93%, 16.96%, 5.71%, and 4.99% than D_40_ during 2017–2018 growing season respectively, while these values for corresponding yield components were 2.79%, 15.71%, 6.11%, and 2.31% during 2018–2019 growing season respectively.

**Table 4:** Interactive effect of lateral spacings and nitrogen application modes on yield components of winter wheat during 2017–2018 and 2018–2019 growing season.

Season	2017–2018				2018–2019			
Treatment	SL (cm)	GS	SPUA (10^4^ ha^-1^)	TGW (g)	SL (cm)	GS	SPUA (10^4^ ha^-1^)	TGW (g)
**D**_**40**_ **N**_**50:50**_	7.92^c^	30.40^d^	492.00^bc^	48.91^cd^	8.48^bc^	35.00^e^	627.00^cde^	50.66^e^
**D**_**40**_ **N**_**25:75**_	8.45^a^	36.90^a^	523.00^a^	51.85^a^	8.62^abc^	41.80^a^	692.00^a^	52.73^a^
**D**_**40**_ **N**_**0:100**_	8.24^ab^	34.10^b^	503.33^ab^	51.60^a^	8.71^a^	39.90^b^	633.33^cd^	52.10^bc^
**D**_**60**_ **N**_**50:50**_	7.88^c^	28.70^e^	487.33^bcd^	48.59^cd^	8.40^c^	32.60^f^	611.67^cde^	49.83^f^
**D**_**60**_ **N**_**25:75**_	8.27^ab^	32.10^c^	511.33^ab^	51.74^a^	8.69^ab^	36.60^c^	671.67^ab^	52.30^b^
**D**_**60**_ **N**_**0:100**_	8.11^bc^	30.60^cd^	491.33^bcd^	51.10^ab^	8.61^abc^	35.30^de^	620.00^cde^	51.68^d^
**D**_**80**_ **N**_**50:50**_	7.29^d^	25.40^f^	466.33^d^	46.81^e^	8.10^d^	31.30^g^	592.00^e^	49.16^g^
**D**_**80**_ **N**_**25:75**_	8.01^bc^	31.20^cd^	490.67^bcd^	49.61^bc^	8.45^c^	35.90^cd^	640.00^bc^	51.85^cd^
**D**_**80**_ **N**_**0:100**_	7.85^c^	27.60^e^	474.67^cd^	48.34^d^	8.53^abc^	31.80^fg^	601.00^de^	50.89^e^
**D**	***	***	**	*	*	***	*	***
**N**	***	***	*	***	**	***	***	***
**D × N**	NS	*	NS	NS	NS	***	NS	NS

Note: SL is spike length, GS is number of grains per spike, SPUA represents number of spikes per unit area, TGW is 1000-grain weight, D = Drip irrigation lateral spacing, N = Nitrogen basal top dressing ratios. Mean values (n = 3) indicating different letters are significantly different at P<0.05. NS stands for non-significant at P<0.05 level. Significance level

*(P < 0.05)

**(P < 0.01)

***(P < 0.001).

As far as NAM is concerned, increasing the top dressed ratio from 50% to 75% significantly improved the yield components but adding all the nitrogen as top dressing in N_0:100_ treatment markedly decreased the yield components than that of N_25:75_ treatment. Averaged across the drip irrigation lateral spacings, N_50:50_ decreased the spike length, number of grains per spike, number of spikes per unit area, and thousand-grain weight by 6.63%, 15.67%, 5.20%, and 5.81% as compared to N_25:75_ in 2017–2018 growing season, and by 3.37%, 13.47%, 8.63%, and 4.62% reduction during 2017–2018 growing season respectively.

### 3.4. Effects of different LS and NAM on ETc and WUE

Data given in Table 5 presents the crop evapotranspiration under different lateral spacing and NAM for the two seasons. No consistent trend in ETc under different lateral spacing was observed during both growing seasons. The average ETc values under D_40_, D_60,_ and D_80_ were 515.63, 520.53, and 496.04 mm respectively during the 2017–2018 season, while these corresponding values during 2018–2019 were 482.93, 485.85, and 495.70 mm respectively. It was noticed that ETc significantly increased with an increase in top dressing ratio. The average values for ETc under N_50:50_, N_25:75_, N_0:100_ were 502.46, 511.58, 518.17 mm, and 475.30, 487.10, 502.08 mm during the growing season of 2017–2018 and 2018–2019, correspondingly.

**Table 5:** Statistics analysis results of ET_c_ (mm) of winter wheat during 2017–2018 and 2018–2019 growing season.

Season	2017–2018				2018–2019			
Treatment	N_50:50_	N_25:75_	N_0:100_	Average	N_50:50_	N_25:75_	N_0:100_	Average
**D**_**40**_	512.76	513.78	520.36	**515.63a**	472.97	480.76	495.04	**482.93b**
**D**_**60**_	511.75	518.84	531.00	**520.53a**	474.97	485.56	497.01	**485.85b**
**D**_**80**_	482.87	502.12	503.14	**496.04b**	477.95	494.99	514.17	**495.70a**
**Average**	**502.46c**	**511.58b**	**518.17a**	**510.73**	**475.30c**	**487.10b**	**502.08a**	**488.16**
**Statistics Analysis Results**	**D**	***			**D**	*		
	**N**	***			**N**	***		
	**D × N**	**			**D × N**	NS		

D = Drip irrigation lateral spacing, N = Nitrogen basal top dressing ratios. Average values indicating different letters are significantly different at P<0.05. Significance level

*(P < 0.05)

**(P < 0.01)

***(P < 0.001).

Water use efficiency was substantially (P < 0.01) influenced by drip irrigation lateral spacings and (P < 0.001) by NAMs during both seasons (Table 6). Increase in WUE was noticed with a decrease in drip irrigation lateral spacing as D_40_ gave higher WUE as opposed to D_60_ and D_80_. It was observed that D_40_ increased the WUE by 6.82%, 8.59%, and by 5.60%, 13.37% than D_60_ and D_80_ during 2017–2018 and 2018–2019 growing season correspondingly. As NAM is concerned, rising the top dressing ratio increased the WUE up to a certain limit and then decreased. Top dressing the 75% of total nitrogen in N_25:75_ improved the WUE by 3.10%, 3.18% and by 5.37%, 7.82% as compared to the N_50:50_ and N_0:100_ during both seasons respectively. Furthermore, the maximum WUE value (1.70 and 1.95) and minimum WUE value (1.51 and 1.64) were observed in D_40_N_25:75_ and D_80_N_50:50_ treatment during both study years respectively.

**Table 6:** Statistics analysis results of WUE (kg m^-3^) of winter wheat during 2017–2018 and 2018–2019 growing season.

Season	2017–2018				2018–2019			
Treatment	N_50:50_	N_25:75_	N_0:100_	Average	N_50:50_	N_25:75_	N_0:100_	Average
**D**_**40**_	1.66	1.70	1.65	**1.67a**	1.88	1.95	1.82	**1.88a**
**D**_**60**_	1.56	1.60	1.53	**1.56b**	1.76	1.85	1.74	**1.78b**
**D**_**80**_	1.51	1.57	1.54	**1.54b**	1.64	1.75	1.59	**1.66c**
**Average**	**1.58b**	**1.62a**	**1.57b**	**1.59**	**1.76b**	**1.85a**	**1.72c**	**1.78**
**Statistics Analysis Results**	**D**		**		**D**		**	
	**N**		***		**N**		***	
	**D × N**		NS		**D × N**		NS	

D = Drip irrigation lateral spacing, N = Nitrogen basal top dressing ratios. Average values indicating different letters are significantly different at P<0.05. Significance level: *(P < 0.05)

**(P < 0.01)

***(P < 0.001).

## 4. Discussion

### 4.1. Effects of LS and NAM on soil moisture and nitrogen distribution

In our study, higher soil moisture contents were observed in D_40_ plots than in D_60_ and D_80_ treatment. This difference might be attributed to dense lateral geometry that allows uniform distribution of moisture. Similar findings have been reported by Chouhan et al. [28] and Gazette [29]. Furthermore, it was noticed that wetted depth was more stable at D_40_ level than that of D_60_ and D_80_ as crop growth behavior under different lateral spacings was different that might have created variation in water distribution. Interestingly, throughout the growing season, it was observed that soil water content in D_80_ reduced earlier than D_40_ and D_60_ indicating short drought stress to plants under D_80_ lateral spacings.

Nitrogen fertilizer applied in the soil had three destinations: plants uptake, remaining in the soil as residual nitrogen, and loss from soil and crop system. The nitrogen loss from the irrigation system may create a serious threat to water receiving bodies [30] and most probably caused a markable increase of nitrate in groundwater [31]. At the winter wheat re-greening stage, we found higher soil nitrogen contents in the deeper soil layer under N_50:50_ treatment. This indicated that at the initial development stage, wheat plants were small and required less quantity of nitrogen fertilizer. Thus, excessive application of basal nitrogen might result in nitrogen eluviation which is the hidden danger of nitrogen loss. Zhao and Si [32] stated that during approximately five months between the sowing and returning green stage, some nitrogen may dissipate through different processes like ammonia volatilization, immobilization, and denitrification by soil microbes. In this study, more nitrogen application as a top dressing in N_0:100_ led to high residual nitrogen in the wheat root zone that was parallel to the findings of Shi et al. [33]. Though the soil moisture and nitrogen residual were more in 60–100 cm soil layer, we could not conclude about no leaching and deep percolation of nutrients beyond the wheat root zone.

### 4.2. Effects of different LS and NAM on crop growth

The impacts of lateral spacings and nitrogen application modes on crop growth were significantly visible in both growing seasons (Figs 6 and 7). In the current study, we found a good response of closer lateral spacing and top dressing all the nitrogen in the form of better plant height, and LAI when compared with other lateral spacings and nitrogen application modes. Widened lateral spacing might create water deficit conditions that led to decrease in crop growth characteristics. Previous studies have also reported a decrease in leaf area caused by water deficit in widened lateral spacing [26, 34]. Water and nitrogen deficiency limits the cell processes like cell elongation and cell division that results in reduction of crop growth [35]. During the early growth stages, N_50:50_ has higher LAI and plant height as compared to the other NAM treatments, but has the least values in later growth stages which further suggests that top dressing more nitrogen in later growth stages is beneficial for winter wheat growth in terms of LAI and plant height.

### 4.3. Effects of different LS and NAM on grain yield

The key concern of the present experiment was to elucidate the most efficient drip irrigation lateral spacing and nitrogen application mode to improve wheat productivity. Our results indicated that grain yield under closer lateral rows was higher than that of the distant lateral spacings. The rise in yield under D_40_ can be explained in terms of high values of yield components in relative treatments. These results corroborate well with Lv et al. [34] findings who showed that yield reduction in widened lateral rows during two consecutive experimental seasons was 9.96% and 8.52% as compared to the closer lateral lines and this reduction was mostly ascribed to reduced grain rate per spike along with 1000-grain weight as observed in our study (Table 4). Mostafa et al. [36] also stated that continuous soil moisture availability in wheat root zone might be responsible for highest values of yield and yield attributes when using double drip irrigation lateral lines rather than single lateral lines. Yield components of wheat showed declined results at D_80_ especially in terms of grains per spike as well as 1000-grain weight which caused reduction in grain yield. These findings are similar to Xu et al. [37] results who stated that grain yield is closely related to the number of grains and spikelets per spike.

In our study, nitrogen application management also played a significant role in yield improvement (Table 3). Our experimental findings showed that appropriate percent of top dressed nitrogen is beneficial for improving winter wheat productivity, which is mainly because of improved 1000-grain weight and number of grains per spike. Although, top dressing of all nitrogen in N_0:100_ treatment is not a feasible strategy for winter wheat. Comparing to N_25:75_, N_0:100_ (top dressed all nitrogen) decreased grain yield by 4.66% and 7.43% in 2017–2018 and 2018–2019 respectively which is further attributed to 15.67% and 13.47% decline in a number of grains per spike, and 5.81% and 4.62% reduction in 1000-grain weight during the growing seasons of 2017–2018 and 2018–2019, correspondingly. Our results are in line with Liu et al. [38] findings where they alluded that decreasing the basal dose and increasing top dressing at the jointing and booting stage significantly improved the yield components and finally the winter wheat grain yield. Furthermore, reduced grain yield under N_0:100_ by applying excessive nitrogen at booting might affect the grain filling and reduced the grain yield by prolonging the growth period and delaying the maturity as reported by Zhang et al. [16] and Liang et al. [39].

### 4.4. Effects of different LS and NAM on ET_c_ and WUE

Generally, there was no consistent trend in ET_c_ of winter wheat during both growing seasons. No significant change was assessed in ET_c_ between 40 and 60 cm lateral spacings, however, there was a difference between 80 cm lateral spacing and D_40_, D_60_ in both seasons. These results are in line with the findings of Chen et al. [26] where he reported no significant effect of lateral spacing on ET_c_. The effects of nitrogen application management on ET_c_ varied under different lateral spacings and the variation among different LS was significant in both seasons. The greater plant growth under N_0:100_ might be the reason for the increment in ET_c_ in this study [40]. Rathore et al. [41] also stated that experimental plots treated with more nitrogen had 8% higher ETc than that of non-fertilized plots.

Generally, the WUE values during 2018–2019 were greater than that of the 2017–2018 season, which could be mainly due to less precipitation during the 2018–2019 season that lowered the total ET_c_. In terms of the decrease in grain yield, the WUE of D_60_ and D_80_ was also lower as compared to the D_40_. This might be due to continuous soil moisture availability in the wheat root zone. Mostafa et al. [36] reported significantly higher values of WUE in double lateral lines as compared to the single laterals. The WUE increased with an increase in the percentage of top dressing of nitrogen up to a certain extent and then tend to decrease, which is in line with findings of Zhang et al. [16] and El-Hendawy et al. [42]. Namely, the wheat plants under 40 cm lateral spacing and N_25:75_ treatment resulted in higher WUE values as compared to the other treatments, which are ascribed to medium crop evapotranspiration and the highest grain yield in this treatment.

## Conclusion

Based on our findings in two years study, the following points may be concluded:

1. Increasing the drip irrigation lateral spacing from 40 to 60 cm and from 60 to 80 cm resulted in lower winter wheat grain yield which is mainly ascribed to the reduction in growth and yield components;
2. Top dressing more nitrogen may improve the growth parameters, but not necessarily increase the grain yield and WUE which indicates that quantifying the optimal nitrogen basal to top dressing ratio is important to gain higher yield;
3. Lateral spacing of 40 cm and NAM of N_25:75_ may be the most suitable combination to gain synchronously greater production of grain and WUE of winter wheat in the NCP.

On the other hand, additional findings are still needed to further explore the movement, distribution, and transformation of irrigated water and applied nitrogen in the soil, and the utilization by wheat plants, and to confirm the applicability of this study findings to other soil and environmental conditions, which will surely be beneficial for sustainable winter wheat production in the NCP.
